# Reactive Oxygen Species Bridge the Gap between Chronic Inflammation and Tumor Development

**DOI:** 10.1155/2022/2606928

**Published:** 2022-06-28

**Authors:** Weihua Yu, Yongmei Tu, Zi Long, Jiangzheng Liu, Deqin Kong, Jie Peng, Hao Wu, Gang Zheng, Jiuzhou Zhao, Yuhao Chen, Rui Liu, Wenli Li, Chunxu Hai

**Affiliations:** ^1^Department of Toxicology, Shanxi Provincial Key Lab of Free Radical Biology and Medicine, Ministry of Education Key Lab of Hazard Assessment and Control in Special Operational Environment, School of Public Health, Fourth Military Medical University, Xi'an, 710032 Shaanxi, China; ^2^Department of Occupational & Environmental Health and the Ministry of Education Key Lab of Hazard Assessment and Control in Special Operational Environment, School of Public Health, Fourth Military Medical University, Xi'an 710032, China; ^3^Student Brigade of Basic Medicine School, Fourth Military Medical University, Xi'an, 710032 Shaanxi, China

## Abstract

According to numerous animal studies, adverse environmental stimuli, including physical, chemical, and biological factors, can cause low-grade chronic inflammation and subsequent tumor development. Human epidemiological evidence has confirmed the close relationship between chronic inflammation and tumorigenesis. However, the mechanisms driving the development of persistent inflammation toward tumorigenesis remain unclear. In this study, we assess the potential role of reactive oxygen species (ROS) and associated mechanisms in modulating inflammation-induced tumorigenesis. Recent reports have emphasized the cross-talk between oxidative stress and inflammation in many pathological processes. Exposure to carcinogenic environmental hazards may lead to oxidative damage, which further stimulates the infiltration of various types of inflammatory cells. In turn, increased cytokine and chemokine release from inflammatory cells promotes ROS production in chronic lesions, even in the absence of hazardous stimuli. Moreover, ROS not only cause DNA damage but also participate in cell proliferation, differentiation, and apoptosis by modulating several transcription factors and signaling pathways. We summarize how changes in the redox state can trigger the development of chronic inflammatory lesions into tumors. Generally, cancer cells require an appropriate inflammatory microenvironment to support their growth, spread, and metastasis, and ROS may provide the necessary catalyst for inflammation-driven cancer. In conclusion, ROS bridge the gap between chronic inflammation and tumor development; therefore, targeting ROS and inflammation represents a new avenue for the prevention and treatment of cancer.

## 1. Introduction

Cancer is one of the most severe diseases affecting humans worldwide owing to its high morbidity and mortality. Over the past 20 years, the number of cancer cases diagnosed each year globally has increased by 50%, reaching 17 million in 2021. Although the survival rate of certain cancers has improved substantially in developed countries, 9 million people die from tumors annually worldwide [1]. Typically, tumorigenesis is attributed to unhealthy lifestyles and environmental pollution [2, 3]. Specifically, increasing physical, chemical, and biological hazards in our living environment contribute to approximately 70–90% of neoplastic diseases [2]. Hence, in recent decades, international research efforts have been dedicated to explaining the role of endogenous and exogenous factors in cancer development.

A link between inflammation response and tumor development has been reported in many epidemiological and experimental studies. In the 19th century, Virchow first observed the presence of large amounts of inflammatory cells in tumors, as well as tumor development at the site of chronic inflammatory lesions [4]. Dvorak et al. also revealed that both tumor masses and inflammatory hyperplasia possess abundant mesenchymal, inflammatory, and angiogenic cells [5]. Moreover, macrophages, which can account for up to 50% of solid tumors, contribute to tumor growth, invasion, and metastasis by releasing various types of cytokines [6–8]. Thus, cancer is also defined as a persistent inflammatory process in which lesions “fail to heal” and invade adjacent tissue [9].

Emerging studies have suggested that continuous exposure to toxic and infectious substances exacerbates inflammatory responses, which may underlie neoplastic progression [10]. Moreover, unhealthy lifestyles characterized by a high caloric intake, insufficient exercise, alcohol consumption, smoking, or stress lead to chronic low-grade inflammation in the human body, a critical risk factor for tumorigenesis [2, 11]. To date, most tumors can be attributed to one or more environmental irritants or unhealthy lifestyle factors, which are also associated with a wide spectrum of chronic inflammatory diseases (Table 1). For instance, alcohol abuse is implicated in chronic hepatitis and hepatocarcinoma [12], *H. pylori* infection can cause chronic gastritis and gastric cancer [13], asbestos-dependent silicosis contributes to lung cancer, patients with gingivitis and periodontitis have a higher risk of oral cancer [14], and long-term UV exposure can lead to dermatitis and skin cancer. In addition, smoking-related bronchitis is associated with lung cancer [15]. In general, 50% of human cancers are related to long-term pathogenic infection and chronic inflammatory diseases [9, 16]. However, the mechanisms by which inflammation drives tumor formation, growth, and metastasis remain unknown.

Environmental irritants and unhealthy lifestyles contribute to impaired redox balance, which causes oxidative damage to proteins, lipids, and DNA [39]. Moreover, oxidative stress and inflammation responses are closely linked to pathophysiological events, which have been implicated in many chronic diseases [40, 41]. In brief, inflammatory cells release a large amount of reactive oxygen species (ROS) and secrete cytokines that also fuel ROS production in adjacent cells. Moreover, ROS regulate several transcriptional genes, further enhancing the expression of proinflammatory cytokines [42]. Many studies suggest that ROS may also enhance genomic instability, malignant cell proliferation, tumor angiogenesis, invasion, and metastasis [43, 44]. Therefore, in this study, we review current research evaluating the potential role and mechanism of ROS in inflammation-induced tumorigenesis.

## 2. Cross-Talk between Oxidative Stress and Inflammation Responses

### 2.1. Redox Balance, ROS Signals, and Their Functions

Redox is a crucial biochemical reaction in living organisms that involves oxidation and reduction. Redox homeostasis plays a key role in maintaining cellular health, whereas a redox imbalance can lead to ROS generation exceeding the ROS-scavenging ability, defined as oxidative stress [45]. To date, several ROS sources have been identified in organisms, such as electron leakage from the electron transport chain (ETC), nicotinamide adenine dinucleotide phosphate oxidases (NOXs), inducible NO synthase (iNOS), and the cytochrome oxidase P450 (CYP450) system. Mitochondrial damage and activation of prooxidant enzymes typically lead to the generation of hydrogen peroxide (H_2_O_2_), superoxide (O^2-^•), hydrogen peroxide (•OH), nitric oxide (NO), and peroxynitrite (ONOO-) [46]. Mitochondrial electron leakage is regarded as the major source of cellular ROS in both physiological and pathological conditions [47]. Many TCA cycle metabolic enzymes are implicated in regulating ROS production, such as succinate dehydrogenase, malic enzyme, and NAPDH oxidase [48, 49]. The intracellular antioxidant defense system, consisting of nonenzymatic antioxidant enzymes (e.g., vitamins (VC and VE), glutathione (GSH), and coenzyme (CoQ)) and antioxidant enzymes (e.g., catalase (CAT), superoxide dismutase (SOD), glutathione reductases (GSTs), heme oxygenase-1 (HO-1), and glutathione peroxidases (GPXs)), is necessary for withstanding oxidative damage [45]. These antioxidant enzymes and GSH are modulated by several redox signaling transcription factors, including Nrf2, PGC-1a, and P53 [46, 50]. Therefore, the ROS generation and antioxidant systems orchestrate the redox status in physiological and pathological conditions. Many reports have shown that various adverse stimuli facilitate oxidative stress by either activating the ROS generation system or impairing the antioxidant system [46, 51]. For example, heavy metal and inhalable particles can result in severe mitochondrial damage and substantial ROS production [52]. Furthermore, participants with high stress, low exercise, alcohol abuse, and an unhealthy diet typically have accumulated oxidative damage [39].

Previously, ROS were regarded as the waste product of metabolism, a trigger for various diseases, and the cause of aging [53, 54]. Excess ROS result in oxidative damage to the major constituents of living cells, including proteins, lipids, and DNA, ultimately contributing to a wide spectrum of pathophysiologies, such as sepsis, aging, obesity, cancer, diabetes, depression, and neurodegeneration [55, 56]. However, emerging evidence indicates that ROS exert many beneficial biological effects through regulating a series of transcriptional and phosphorylation processes [45, 57, 58]. For instance, ROS not only maintain the cell cycle and division but also play a key role in tumor chemotherapy and radiotherapy [59, 60]. In general, intracellular ROS levels determine biological outcomes (Figure 1), whereby low ROS levels are associated with regulating cell proliferation, differentiation, and malignant transformation, whereas high ROS levels directly cause cell apoptosis or necrosis [45]. Patients with acute poisoning, infection, and irradiation exposure typically exhibit large-scale ROS production and apoptotic cells throughout the body, whereas patients with tumor and chronic inflammatory diseases typically exhibit low-grade oxidative stress and abnormal cell proliferation in lesions [51]. Moreover, Wang and Hai and Meng et al. implied that the specific species, application times, and intracellular spaces of ROS/reactive nitrogen species (RNS) determine their biological functions [46, 61]. Although many studies have assessed ROS levels in different disease models, systematic analysis of ROS dynamics in pathological conditions is still lacking. To date, there is no effective method for detecting ROS levels in clinical applications. Therefore, the redox network in organisms is highly complex, and redox homeostasis is crucial for maintaining human health. However, the precise evaluation of the redox status in the human body is still in its infancy, limiting the use of antioxidants in disease prevention and treatment.

### 2.2. Inflammation Response and Regulatory Network

Inflammation is the most common pathophysiological process, characterized by the accumulation of inflammatory cells, cytokines, and chemokines. There are many sources of inflammation, including physical, chemical, biological, and unhealthy lifestyle factors, as well as chronic and autoimmune diseases [62] (Table 2). According to the duration of inflammation, the inflammation process can be divided into acute and chronic stages. Acute inflammation is typically characterized by a sudden onset, a short duration, the presence of exudative lesions, and granulocyte infiltration. Conversely, chronic inflammation may last months to years and is often dominated by hyperplasia lesions, characterized by macrophage and lymphocyte infiltration [63]. Once an organism senses infection or trauma, acute inflammation is triggered, becoming the key mechanism by which the innate immune system removes pathogens [64]. However, excessive immune system activation may result in cytokine storms, sepsis, and subsequent multiple organ dysfunction, the major cause of death in clinical emergencies [65]. If the irritations persist, aggregation of inflammatory cells and cytokines can transform acute inflammation into the chronic stage, potentially inducing local and systemic deleterious effects [62]. Many studies have revealed that uncontrolled low-grade inflammation is a direct cause of chronic diseases, including obesity, diabetes, cancer, nonalcoholic fatty liver disease, and neurodegenerative diseases [65, 66]. Moreover, chronic systemic inflammation leads to more than 50% of disabilities and deaths worldwide. Therefore, targeting the immune system has become an effective therapeutic strategy for cancer and other inflammatory diseases. Hundreds of natural and synthetic anti-inflammatory drugs that have successfully cured large numbers of patients are currently available [67]. Recently, the link between chronic inflammation and tumorigenesis has garnered substantial attention [42, 68]. That is, many tumors arise from sites of chronic irritation, infection, and inflammation [69], and inflammatory cells within the tumor microenvironment (TME) are indispensable for modulating the neoplastic process [9]. However, despite notable progress in this research field, how chronic inflammation induces tumor formation remains unclear. Thus, elucidating this mechanism can contribute to the prevention and treatment of cancer.

Various inflammatory cells are involved in acute and chronic pathologies. During sepsis, countless immune cells (such as neutrophils and macrophages) can be recruited to fight infection, resulting in the uncontrolled initiation of cytokine cascades [87, 88]. Compared to nonobese subjects, patients with obesity contain more macrophages in their adipose tissues; these cells undergo proinflammatory differentiation, leading to low-grade inflammation and insulin resistance [89]. Notably, inflammatory cells, such as macrophages, lymphocytes, neutrophils, mast cells, and immature myeloid cells, are core components of the TME [8, 90]. Once activated, these cells release a large range of cytokines and chemokines, including tumor necrosis factor-*α* (TNF-*α*), interleukin- (IL-) 6, interferon-*γ* (IFN-*γ*), NO, monocyte chemotactic protein-1 (MCP-1), and chemokine ligand 10 (CXCL10), which in turn boost the recruitment of inflammatory cells to lesions [88]. To date, several transcriptional signaling pathways that modulate the onset of inflammatory signaling cascades have been identified. For example, TLR4 is the ligand of bacterial endotoxins (lipopolysaccharides, LPS), which plays a critical role in activating macrophages and dendritic cells. Moreover, LPS, IFN-*γ*, and TNF-*α* promote the activation of nuclear factor *κ*-B (NF*κ*B), the signal transducer and activator of transcription (STAT), inducible nitric oxide synthase (iNOS), activator protein-1 (AP-1), hypoxia-inducible factor-1*α* (HIF1-*α*), cyclooxygenase-2 (COX-2), and NOD-like receptor protein 3 (NLRP3) inflammasome [91, 92]. Inhibition of these transcriptional factors hinders the production of inflammatory mediators and cytokines [91]. Targeting the transcription of inflammatory networks can provide new therapeutic strategies for various chronic diseases, including cancer.

### 2.3. Relationship between ROS Signals and Inflammation

Recent research has revealed the relationship between ROS signaling and inflammation responses. Briefly, oxidative stress and inflammation mutually interact in a feedback loop (Figure 2). On the one hand, inflammatory cells and associated cytokines often contribute to redox imbalances in infectious and cancerous lesions. Evident DNA oxidative damage is typically observed in hepatocytes and lung epithelial cells coincubated with activated neutrophils [93]. In response to infection and trauma, respiratory burst is activated in neutrophils and macrophages, generating large amounts of ROS and RNS, which are crucial for defense against invading pathogens. Proinflammatory cytokines also boost ROS accumulation in both phagocytic and nonphagocytic cells, leading to oxidative stress in various acute and chronic diseases [94, 95]. Moreover, LPS, IFN-*γ*, and TNF-*α* stimulation leads to proinflammatory differentiation of macrophages and abundant ROS production. On the other hand, cellular redox signaling plays a critical role in regulating the inflammatory response. ROS accumulation contributes to macrophagic proinflammatory differentiation and cytokine secretion, while ROS reduction promotes anti-inflammatory differentiation of macrophages and inflammation resolution [94]. For example, Yu et al. found that mitochondrial fission-dependent ROS production is required to activate NF*κ*B in differentiated proinflammatory macrophages [96]. Zhou et al. found that mitophagy inhibition boosts the NLRP3 inflammasome by inducing mitochondrial damage and ROS generation [97]. ROS also foster the transcriptional activation of abundant proinflammatory cytokines through the activation of iNOS, COX-2, and STAT3 signaling pathways, whereas antioxidants can curtail these processes [95]. Substantial evidence showed that increased DNA damage and mutation rates were observed in the inflammatory microenvironment. Oxidized mtDNA can drive the assembly of the NLRP3 inflammasome, which contributes to the development of chronic inflammation and associated diseases [98]. Lipid oxidation is also tightly linked to inflammation responses. Briefly, low-density lipoprotein oxidation induces activation of inflammatory cells, whereas high-density lipoprotein (HDL) exhibits prominent antioxidant and anti-inflammatory properties [95]. Furthermore, ROS-dependent necrotic cell death exacerbates inflammation response by recruiting abundant macrophages and neutrophils into lesions. In contrast, clearance of ROS-induced apoptotic cells by macrophages contributes to the resolution of inflammation [83, 99]. Therefore, inflammation and oxidative stress occur simultaneously and are closely linked to pathophysiological processes, whereby one is easily stimulated by the other. In brief, an increase in inflammatory cell-derived ROS exacerbates inflammation, and ROS-dependent inflammation leads to secondary oxidative stress, forming a vicious circle [100]. Notably, inflammation onset and redox signaling are regulated by independent pathways. The intracellular redox status is determined by the ROS-generating and ROS-scavenging systems, whereas the inflammation response is modulated by several inflammatory transcriptional factors, especially NF*κ*B [95]. Therefore, antioxidant agents or inflammatory drugs alone can only partially improve oxidative stress and inflammation without fully eradicating the problem. Combined administration of anti-inflammatory agents and antioxidants may be a helpful approach to address acute and chronic inflammatory damage.

## 3. Changes in Redox and Inflammatory States during Neoplasia

Recent literature lists 10 key hallmarks of cancer, including genome instability, uncontrolled proliferation, evasion of growth suppression, immune escape, immortality potential, tumor-promoting inflammation, deregulated metabolism, angiogenesis, invasion, and metastasis [101]. It is no doubt that inflammatory cells and associated cytokines play a crucial role in regulating cancer development. Solid tumors comprise distinct phenotypic cell populations, ranging from neoplastic cells, nonmalignant stromal cells, migrating hematopoietic cells, and various immune cells. Elevated ROS in tumor masses endows malignant cells with the ability to proliferate rapidly, avoid programmed cell death, migrate, and invade [42, 44, 102]. Moreover, the increased ROS in TME affects angiogenesis as well as the survival and function of nonmalignant stromal cells and immune cells [103]. Therefore, most of these hallmarks are tightly linked with ROS signaling; targeting the redox system may directly determine the survival and death of cancer cells [102, 104, 105]. In the next section, we introduce the changes in redox and inflammatory states during tumorigenesis.

### 3.1. Redox Fluctuations and Their Functions in Tumors

Many studies have shown that cancer cells possess higher levels of ROS than normal cells, which play a vital role in regulating tumor initiation, promotion, and progression [42, 44, 106]. In clinical specimens from patients with cancer, the ROS level is much higher in tumor masses than in paracancerous tissues, or in equivalent specimens from healthy individuals [107]. Interestingly, ROS reportedly play a dual role in tumor development and treatment. On the one hand, increased ROS levels endow tumor cells with more survival advantages through regulating metabolism, proliferation, and angiogenesis. On the other hand, ROS are also a powerful weapon for suppressing or killing cancer cells, which plays a crucial role during chemotherapy and radiation therapy. ROS-dependent apoptosis, ferroptosis, parthanatos, and autophagy-mediated cell death have been proved to suppress tumor growth through regulating GPXs, SLC7A11, and PARP-1 [108–111]. Moreover, several pathways have been confirmed to stimulate ROS generation in tumor cells. Substantial evidence showed that mitochondria are the major sources of ROS in both oncogene- and damage-related carcinogenesis [112]. Mitochondrial structure and function in malignant cells differ from those in normal cells, exhibiting increased fission, shortened morphologies, reprogramed metabolism, and reduced ATP generation, ultimately promoting increased electron leakage and ROS generation [47]. Moreover, inhibition of mitochondrial fission can impair ROS generation and cell proliferation in Ras-driven cancer [113]. Damaged DNA also hinders oxidative phosphorylation and ROS release in mitochondria. Moreover, NOX4 activation and ER stress lead to increased ROS in cancer cells, which play a key role in regulating tumor cell hyperproliferation [111]. Many studies have revealed that oncogenes are implicated in increased ROS production. Myc inhibits PGC-1*α* expression and mitochondrial biogenesis, resulting in ROS accumulation [114]. The knockout of p53 in A549 carcinoma cell lines can also increase ROS by blocking the expression of several antioxidant genes, such as SOD2 and GPX1 [115]. Moreover, inflammatory cells and associated cytokines contribute to disrupting redox balance in tumor cells [116]. Accumulation of ROS and DNA damages are observed in hepatocytes coincubated with neutrophils, macrophages, and TNF-*α* [117, 118].

Furthermore, the expression of Nrf2 and related antioxidant enzymes in tumor cells is much higher than that in normal cells [104, 105, 119]. Nrf2 is traditionally regarded as a potent tumor suppressor by reducing exogenous and endogenous ROS. Generally, Nrf2 is directly or indirectly involved with most cancer hallmarks, such as carcinogenesis, aberrant proliferation, evasion of apoptosis, metabolic reprogramming, imbalanced redox, sustained angiogenesis, metastasis, and therapy resistance [104]. Nrf2 knockdown or inhibition may increase the potential for neoplasia in animals stimulated with various carcinogens [105]. However, recent evidence has shown that persistent Nrf2 activation exerts harmful effects in patients with cancer. That is, Nrf2-induced antioxidant enzymes drive metabolic reprogramming and redox homeostasis, fueling cell proliferation and tumor growth [105]. Inhibition of GPX1 activity and GSH synthesis are also associated with reduced proliferative capacity in various tumor cells [120, 121]. However, increased Nrf2 signaling facilitates tumor-cell resistance to radiotherapy and chemotherapy by enhancing their ability to eliminate excessive ROS. Patients with high Nrf2 and GSH levels in tumor cells typically exhibit malignant phenotypes implicated in tumor metastasis and poor prognoses [104, 121]. Hence, the Nrf2-related antioxidant system may play a double-edged role in tumor development.

Here, we compared the redox homeostasis in normal and cancer cells (Figure 3). Tumor cells inherently produce a higher level of ROS than normal cells, including H_2_O_2_, O^2-^•, •OH, and NO. The increased ROS in malignant cells originated from mitochondrial ETC, aberrant metabolism, activation of oncogenes, inactivation of tumor suppressor genes, and inflammatory stimuli [45]. To counter the oxidative damage, cancer cells deploy a more robust antioxidant system through the activation of Nrf2 and its target genes, such as GPX1, CAT, GSH, SOD_1_, SOD_2_, and HO-1 [104, 105, 122]. Thus, both normal and malignant cells maintain cellular redox homeostasis by regulating ROS production and elimination; however, higher-level redox signaling endows cancer cells with greater survival potential.

### 3.2. Role of Inflammatory Status Changes in Tumorigenesis

The immune system of organisms has a vital role in carcinogenesis and its treatment. In general, adaptive immunity acts as a suppressor of cancerization by immunosurveillance, whereas innate immunity often contributes to the neoplastic process [123]. Recent studies have shown that most solid tumors contain large numbers of inflammatory cells, including T cells, macrophages, neutrophils, and immature myeloid cells. Still, their role in tumor progression remains complex and controversial [68, 124]. Cytotoxic CD8^+^ T cells can directly kill tumor cells, reportedly the most powerful weapon for cancer immunotherapy [125, 126]. CD4^+^ helper T cells (Th), such as Th1, Th2, and Th17, also affect CD8^+^ T cell proliferation and cytotoxicity by secreting a series of inflammatory cytokines [127]. Notably, FasL and PDL-1 in TME contribute to the apoptosis and exhaustion of CD8^+^ T cells, which results in tumor immune escape [126]. Encouragingly, genetically engineered T cells, tumor-infiltrating lymphocytes, and CAR-T cells have been widely used in tumor immunotherapy, bringing hope to patients with cancer [128]. In addition, immature myeloid cells are abundant in cancer patients as well as in mouse models, which is conducive to immune escape and tumor metastasis [129]. Neutrophil accumulation in TME, regarded as a biomarker of poor clinical outcomes in various cancers, also contributes to cancer initiation, promotion, and progression [130]. Deleting hepatic neutrophils with specific antibodies alleviates DNA damage and hepatocellular carcinoma in diethyl nitrosamine- (DEN-) treated mice [117]. Interestingly, macrophages have a bidirectional regulatory role in coordinating immune responses, which can hinder or foster the efficiency of cancer immunotherapies [131]. M1 phenotype macrophages, which can directly kill tumor cells or indirectly activate other antitumor immune cells such as T cells and NK cells, are abundant during the initial tumor stages [6, 132]. Conversely, TME is characterized by abundant M2 phenotype macrophages, termed tumor-associated macrophages (TAMs), which play a critical role in regulating tumor initiation, angiogenesis, invasion, and chemoresistance [7, 133]. Moreover, TAMs are involved in suppressing T cell-induced antitumor immunity, and the specific depletion of CD163^+^ TAMs induces massive infiltration of activated T cells and tumor regression [134]. TAMs also facilitate tumor-cell growth and angiogenesis by generating various types of growth factors, including transforming growth factor-*β* (TGF-*β*), epidermal growth factor (EGF), and vascular endothelial growth factor (VEGF) [7, 135, 136]. Therefore, immune dysfunction is a hallmark of cancer, and targeting these inflammatory cells contributes to preventing and treating tumors.

Furthermore, recent reports have shown increased inflammatory cells in the blood of patients with cancer. Indeed, circulating lymphocytes, neutrophils, and myeloid-derived suppressor cells (MDSCs) are recognized as useful prognostic and predictive markers for various types of tumors [137, 138]. Emerging evidence suggests that a high count of circulating neutrophils is a strong prognostic factor for the survival of patients with various cancers [130]. The accumulation of CD4^+^ and CD8^+^ T cells, which fuels cancer growth and metastases, can be used to predict the prognosis of cancer patients [139]. Moreover, MDSCs refer to a heterogeneous population of early myeloid cells, comprising naïve granulocytes, macrophages, and dendritic cells at distinct stages of differentiation. Compared with healthy volunteers, the number of circulating MDSCs is much higher in cancer patients, especially those with melanoma, gastrointestinal cancer, and breast cancer [140]. MDSCs can inhibit NK cell-mediated cytotoxicity and CD8^+^ T cell-induced immune adaptations. An increasing white cell count and neutrophil to lymphocyte ratio are also independent predictors of poor outcomes in patients with lung cancer [141].

## 4. ROS Play a Vital Role in Inflammation-Induced Cancer

It is now widely accepted that chronic inflammation is implicated in various steps of carcinogenesis, such as cell malignant transformation, proliferation, migration, and resistance to chemotherapy and radiotherapy [9, 69, 142, 143]. In addition, ROS have been recognized as important contributors in the development of various types of cancer (Table 3). Here, we discuss the potential role and mechanisms underlying ROS signaling involvement in the inflammation-associated neoplastic process.

### 4.1. ROS Drives Inflammation-Induced Genomic Instability

Genomic instability is a hallmark of cancer cells and the origin of malignant transformation. In hereditary cancers, mutations in DNA repair genes cause genomic and chromosomal instability, which further drives cancer development. In nonhereditary cancers, environmental irritants and unhealthy lifestyle factors induce DNA damage and gene mutations. Therefore, increased genomic stability is crucial for the development of carcinogen-induced cancer [153]. The link between inflammation and genomic instability in carcinogenesis has been confirmed by numerous studies [154]. For instance, coculture with activated macrophages and neutrophils causes genetic damage in normal cells, including DNA strand breaks, sister chromatid exchanges, and mutations [117, 154]. Neutrophils can lead to DNA damage accumulation by activating procarcinogens such as aflatoxins, benzopyrene, and quartz particles [155, 156]. LPS also amplifies aflatoxin hepatotoxicity in a TNF-*α*-dependent manner [157]. Increased inflammatory cells and DNA damage are typically observed in patients with periodontitis and gingivitis [158]. Moreover, as a product of nitrative DNA damage, 8-nitroguanine is enhanced in clinical specimens from patients infected with tumor-related pathogens, including human papillomavirus, *Helicobacter pylori*, hepatitis B virus, and Epstein–Barr virus [158, 159]. Interestingly, DNA oxidative damage and mutations typically occur at sites of tumorigenesis induced by infections or asbestos exposure [118, 160]. Thus, inflammation-induced DNA damage and genomic instability play a critical role in the initiation of tumors.

Since the 1990s, several reports have pointed to ROS as the major driving force of DNA damage and genomic instability during the neoplastic process [161]. For example, ectopic expression of oncogenic Ras induces the ROS-dependent malignant transformation of human fibroblasts. The mutation or knockdown of tumor suppressor p53 contributes to increasing ROS and DNA oxidation, indicating the antioxidant function of p53 [162, 163]. Dietary supplementation with N-acetyl-L-cysteine (NAC) impairs the development of lymphomas in p53-knockout mice and the growth of p53-deficient cancer xenografts [115]. Moreover, 8-hydroxydeoxyguanosine (8-OHdG), 8-nitroguanine, *γ*H2AX, and 4-hydroxynonenal (4-HNE) are sensitive biomarkers of nitrative and oxidative DNA damage, which contribute to genomic instability [44]. Additionally, the •OH radical is the most reactive ROS, which can attack the ring structure of guanine in DNA, forming 8-OHdG. In general, more oxidative DNA adducts correspond to a greater risk of carcinogenesis. Recent evidence has revealed the link between environmental carcinogens and DNA oxidative damage, whereby abundant 8-OHdG and 4-HNE were observed in the urine of patients suffering from radiation. In addition, phorbol 12-myristate 13-acetate (PMA) and UV exposure led to 8-OHdG accumulation in the skin of animals [164, 165]. Moreover, mice treated with the carcinogen DEN exhibited elevated ROS, 4-HNE, and *γ*H2AX in their hepatic tissues, which can be reduced by dietary antioxidant butylated hydroxyanisole [117]. Therefore, ROS are a major cause of genomic instability in both hereditary and nonhereditary cancers.

According to many studies, most inflammation-induced DNA damage and genomic mutations are associated with ROS and RNS (Figure 4) [142, 166]. For instance, mice with inflammatory bowel disease exhibit ROS-dependent accumulation of 8-OHdG in colon epithelial cells [167, 168]. In DEN-treated mice, the accumulation of hepatic neutrophils stimulates hepatocellular ROS generation and telomere DNA damage, which is ameliorated by antioxidant agents [117]. Asbestos-induced inflammatory cell infiltration enhances ROS/RNS generation, further contributing to DNA damage in adjacent epithelial cells [169, 170]. Numerous reports also reveal that DNA damage can exacerbate inflammatory development, ultimately leading to the accumulation of DNA damage [118, 171]. The cross-talk between DNA damage and inflammation exerts a critical role in cancer, depression, neurodegeneration, and cardiovascular diseases [118, 142, 166, 168]. DNA damage can also result in mutations and genomic instability without efficient repair, which underlies the malignant transformation of cells. Interestingly, emerging evidence has revealed that ROS/RNS can disrupt DNA repair pathways, including base excision repair (BER), direct reversal, and double-strand break repair [142, 172–174]. Patients with cancer exhibit lower BER efficiency than healthy participants, partially due to the ROS-dependent inhibition of DNA repair enzymes. Moreover, cytokine-induced NO production can inhibit several DNA repair proteins [175]. DNA nitrative damage is predominantly repaired by the 8-oxoguanine glycosylase- (OGG1-) related BER pathway, and S-nitrosylation of OGG1 leads to reduced OGG1 activity [176, 177]. Notably, the overdose accumulation of ROS promotes DNA damage and causes cell apoptosis rather than malignant transformation [178, 179]. Therefore, low-grade ROS generation during chronic inflammation contributes to genomic instability by inducing DNA damage and impairing DNA repair.

### 4.2. ROS Causes Hyperproliferation in Malignant Cells

The potential for uncontrolled proliferation is the greatest difference between malignant and normal cells and an important feature in cancer. The involvement of ROS as secondary messengers in the regulation of cell proliferation has been well documented [45]. *In vitro* stimulation with H_2_O_2_ leads to increased viability and proliferation of native hepatocytes and tumor cells, whereas the inhibition of H_2_O_2_ blocks fetal hepatocyte proliferation and liver regeneration [180, 181]. Moreover, mitochondrial nitric oxide is critical in regulating cell proliferation during animal liver development [182]. Overexpression of catalase delays serum-induced cell proliferation in endothelial cells, and the catalase inhibitor impairs this process, indicating that endogenously produced H_2_O_2_ is necessary for cell division [183]. Furthermore, cancer cells typically possess higher ROS levels than normal cells, which is critical for sustaining their unlimited replicative ability. In Ras-driven cancer cells, abnormal mitochondria and activated NOX4 boost ROS-dependent cell proliferation [184]. The inhibition of mitochondrial fission can hinder ROS generation and subsequent cell proliferation in hepatocellular carcinoma cells [185]. H_2_O_2_ is also necessary for maintaining increased proliferation in breast tumor cells [106]. Wang Z et al. proved that aloin inhibits gastric cancer cell proliferation by blocking the NOX2-ROS-Akt signaling pathway [186]. Additionally, Diao et al. demonstrated that vitamin E could promote breast cancer cell proliferation by inhibiting ROS production and p53 expression [187]. Paradoxically, the inhibition of GSH and GPX1 results in higher levels of ROS, which may impair cell proliferation and even trigger cell apoptosis [120, 188].

The eukaryotic cell cycle is crucial for DNA replication and cell proliferation, and its disruption leads to oncogenesis. Various studies have suggested that ROS signaling is involved in driving cell cycle progression from quiescence (G_0_) to proliferation (G1, S, G2, and M) and back to quiescence [45, 51, 58]. Intracellular ROS levels exhibit regular fluctuations in different phases of the cell cycle. ROS are generally maintained at low levels during the G_0_/G_1_ phase before gradually increasing as the cell cycle progresses, peaking in the M phase, and then returning to lower levels at the end of cell division [102]. The cell cycle is controlled by several cyclins and cyclin-dependent kinases (CDKs). Inhibition of ROS blocks serum-induced G0/G1 to S phase transition by reducing the activities of cyclin E-CDK2 and cyclin D-CDK4 complexes [183, 189, 190]. Catalase is known as an H_2_O_2_ scavenger; catalase overexpression yields decreased CDK activities and an extended G_0_/G1 phase, indicating that endogenously generated H_2_O_2_ is necessary for cell proliferation [183]. Studies also show that ROS are implicated in modulating CDK inhibitors, including p21, p27, and p53 [58, 190]. Moreover, mitogen-activated protein kinase (MAPK) is a key redox-sensitive pathway crucial for cell proliferation. Reportedly, ROS promote serum-induced cell proliferation and hepatic regeneration in liver-resected mice via the activation of extracellular regulated protein kinases (ERK), c-Jun N-terminal kinase (JNK), and p38 subfamilies [180, 191]. Protein kinase C (PKC) and PI3K-Akt pathways also play a key role in EGF-induced cancer cell proliferation and migration in ROS-dependent pathways [192].

Moreover, emerging evidence emphasizes the critical role of inflammation-derived ROS in modulating the aberrant proliferation of malignant cells. TAMs are the dominant components of TME, which can secrete large amounts of cytokines (IL-6 and IL-10) and growth factors (EGF and VEGF). Zhang et al. proved that TAM-generated TGF-*β* enhances the survival and proliferation of colorectal cancer cells [136]. Moreover, IL-10 secreted by TAM regulates proliferation and invasion in gastric cancer cell STAT3 signaling [193], and IL-6 stimulation promotes the increased proliferation of cancer cells [194]. Interestingly, ROS plays a critical role in the proliferation of cancer cells induced by EGF and VEGF by activating MAPK and PKC pathways [195, 196]. Therefore, higher ROS are associated with the aberrant proliferation of tumor cells through various pathways (Figure 5).

### 4.3. Inflammation and ROS Fuel Tumor Metastasis

Tumor metastasis is the dominant cause of most cancer mortality, which is also a complex and multistep process, including migration, invasion of tumor cells, and angiogenesis around tumor lesions [197]. Clarifying the mechanisms involved in tumor metastasis is critical for improving the survival rate of cancer patients. Many reports have shown that most tumor metastasis arises from the spread of inflammatory lesions [198]. Chronic inflammation contributes to the progression of tumor metastasis by secreting a range of growth factors, cytokines, and chemokines [143]. Inflammatory cells in the TME promote cancer cell metastasis through the release of several adhesion molecules and chemokines, such as intercellular cell adhesion molecule-1 (ICAM-1) and matrix metalloproteinases (MMPs) [143, 199]. Epithelial-mesenchymal transition (EMT) refers to the biological process of epithelial cells transforming into mesenchymal-like cells, which is involved in inducing chronic inflammation and cancer metastasis [200]. Emerging evidence has revealed the cross-talk between chronic inflammation and EMT programs [201]. Macrophages and related cytokines play a vital role in promoting EMT formation, leading to the generation of various proinflammatory cytokines in cancer and pathologic cells [201]. Furthermore, therapies targeting inflammatory cells can attenuate the metastasis of various types of cancer. Moreover, many studies show that inflammation is implicated in angiogenesis, which is critical for various neoplastic conditions [143, 202]. TAM infiltration also contributes to tumor angiogenesis by producing a series of proangiogenic growth factors. Additionally, various inflammatory cytokines and pathways, such as COX2, IL-8, IL-22, and CXCR-2, are involved in promoting angiogenesis and subsequent tumor invasion and lymph node metastases [202].

Growing evidence indicates the critical role of ROS in modulating the various steps of cancer metastasis [44, 103]. Excessive ROS induce tumor invasion by elevating the possibility of malignant cell migration. MMPs and ICAM-1 are master regulators that sustain the migration properties in various cancer types. Moreover, IL17A stimulates esophageal adenocarcinoma cell invasion via ROS-NF*κ*B-dependent MMP-9 activation [203], and H_2_O_2_ promotes the invasion of colon cancer cells by augmenting MMP-7 expression [204]. NOX-mediated ROS play a critical role in modulating cancer cell migration by increasing the expression and activity of MMPs, which can be blocked by a series of antioxidant agents [205, 206]. Neutrophils also promote the ROS-dependent expression of ICAM-1 in inflammatory lesions and tumor masses [207]. Furthermore, ROS accumulation has been observed during the EMT of TGF-*β*-induced cancer cells [208]. Inhibition of ROS generation via the targeting of mitochondria and NOX4 blocks EMT progression and metastasis in various cancers. ROS reportedly trigger EMT by activating various pathways, including E-cadherin, N-cadherin, vimentin, and Snail [209]. Moreover, the Nrf2 level negatively correlates with the abundance of TGF-*β*, EMT, and cell migration in patients with lung cancer [210]. Many antioxidant agents, including curcumin, resveratrol, and CoQ10, can inhibit the aggressive metastatic phenotype of malignant tumor cells by targeting EMT [211]. However, ROS also facilitate angiogenesis programs, which are indispensable for solid tumor growth and metastasis [212]. NOX- and mitochondria-derived ROS are also crucial for VEGF-induced angiogenesis [213]. ROS also promote tumor angiogenesis and invasion by modulating the hypoxia-inducible factor (HIF-1) [209]. Furthermore, H_2_O_2_ can directly cause endothelial injury at high concentrations (>125 *μ*M), as well as stimulate angiogenesis at low concentrations (0.1–10.0 *μ*M) [214, 215]. Finally, the Nrf2 signaling pathway and several antioxidant agents can inhibit angiogenesis in several types of cancer [216]. Thus, ROS neutralization is beneficial for inflammation-related tumor metastasis.

### 4.4. ROS Foster Tumor-Cell Survival and Therapy Resistance

Tumor cells exhibit a greater survival ability than normal cells by avoiding apoptosis, which is also a hallmark of cancer. Reportedly, ROS can control the survival and death of tumor cells according to their intracellular concentration [42, 217]. Indeed, slightly higher ROS in the TME are beneficial for tumor-cell survival. Akt, a well-known serine-threonine kinase, is critical for enhancing tumor-cell survival via the phosphorylation and inactivation of several proapoptotic genes, including Bad, Bax, and caspase 9 [217]. Shearn et al. proved that 4-hydroxynonenal reduces cell survival in hepatocellular carcinoma by inhibiting H_2_O_2_-dependent Akt activation [181]. Moreover, the inhibition of NOX-mediated ROS generation leads to cell apoptosis by promoting the inactivation of the Akt signaling pathway in oral squamous cell carcinoma [218]. Many studies have reported that p53 is implicated in triggering DNA repair and cell apoptosis. The mutation of p53 typically leads to increased basal ROS levels in tumor cells, impairing apoptosis and enhancing survival [219, 220]. Tumor cells deficient in wild-type p53 display greater survival ability in response to radiation and toxic chemicals [219]. However, evidence suggests that excessive ROS induce cell apoptosis by modulating various signaling pathways. Furthermore, a higher concentration of ROS can induce p53 activation and cell apoptosis in a mitochondrial-dependent and -independent manner [221, 222]. Irritant-induced excessive ROS levels also lead to cell apoptosis by modulating the PI3K/Akt pathway [223, 224].

Radiotherapy and chemotherapy are widely used treatments for various lymphoma and solid tumors. In fact, radiation and multiple drugs kill tumor cells by inducing ROS overdose and subsequent cell death [225]. However, cancer cells can acquire radioresistance and chemoresistance during therapy, which is a key reason for poor prognosis in oncology treatment. One of the most important features of therapy-resistant cancer cells is their higher antioxidant capacity compared to that of normal and nonresistant cancer cells [42]. Growing evidence suggests that ROS-induced resistance in cancer cells modulates several redox-sensitive transcription factors such as Nrf2, NF*κ*B, and HIF-1*α* [225]. Recently, targeting the Nrf2-related antioxidant system in the TME has been regarded as an effective approach for killing therapy-resistant cancer cells. For example, Singh et al. found that a small molecule inhibitor of Nrf2 (ML385) effectively reverses chemotherapeutic resistance in non-small-cell lung cancer [226]. Ge et al. and Chen et al. proved that iASPP, a new antioxidant agent, can drive drug resistance in cancer cells by competing with Nrf2-Keap1 binding [227, 228]. Xu et al. revealed the critical role of PAQR4 in promoting chemoresistance in non-small-cell lung cancer by blocking Nrf2 protein degradation [229]. Many studies have also emphasized the critical role of GSH and GPX-1 in the development of cancer resistance [188]. Furthermore, activation of the transcription factor NF*κ*B is linked to tumor-cell resistance induced by several chemotherapeutic agents. Cytokines and ROS in the TME can promote NF*κ*B overexpression in cancer cells, further increasing cell survival and radioresistance [230, 231]. Moreover, HIF-1*α* is associated with both inflammation and tumor therapy resistance. Dong et al. found that ROS can activate metabolic reprogramming and 5-fluorouracil resistance in colorectal cancer by inducing the HIF-1*α* signaling pathway [232]. Lamberti et al. showed that activation of the ROS-Erk1/2-HIF-1 axis contributes to tumor-cell resistance to photodynamic therapy [233]. Therefore, these findings reveal that increased ROS and antioxidant ability in the TME are vital for inducing survival and tumor therapy resistance.

Inflammatory cells and cytokines in the TME also play a crucial role in driving tumor-cell survival and therapy resistance. TAMs, the dominant immune cells in the TME, contribute to cancer chemotherapy resistance by releasing survival factors or activating antiapoptotic programs in malignant cells [234, 235]. For instance, breast cancer cells cocultured with macrophages exhibit therapy resistance to paclitaxel, which is related to Akt pathway activation, or produce TGF-*β*, VEGF, and IL-10 [236, 237]. Pyrimidine, cholesterol, IL-6, and exosomal miRNA released by TAMs are also associated with enhanced therapy resistance in various cancer cells [238–240]. Moreover, the role of ROS in inflammation-associated chemotherapy has been revealed by many studies. For instance, Xia et al. showed that TNF-*α* stimulation boosts hepatocellular carcinoma proliferation and resistance to apoptosis by inducing ROS-dependent HIF-1*α* [241]. Moreover, an *in vivo* study showed that the ROS-HIF-1*α* signaling axis is necessary for chemoresistance induced by multinucleated cells by secreting VEGF [242]. The ROS/JNK pathway is also implicated in chaetocin-mediated colorectal cancer cell apoptosis and macrophage enhancement [243]. Furthermore, the ROS-dependent activation of the NLRP3 inflammasome contributes to 5-fluorouracil resistance in oral squamous cell carcinoma [244]. Thus, increased ROS in tumor cells explains the relationship between chronic inflammation and chemotherapy resistance.

## 5. Antioxidants and Anti-inflammatory Agents in Tumor Therapy

Recently, substantial progress has been made in treating cancer patients, including surgical removal, chemotherapy, radiotherapy, and immunotherapy. However, high cell motility and cancer recurrence rates remain a serious problem for oncology patients. Here, we discuss recent advances in applying antioxidants and anti-inflammatory agents to cancer prevention and therapy.

### 5.1. Anti-inflammatory Drugs for Cancer Prevention and Treatment

As a hallmark of cancer, inflammation plays a key role in each step of neoplasia. Although the last decade has witnessed the successful application of immunotherapies for cancer, the role of anti-inflammatory drugs in cancer therapy remains uncertain. Here, we summarize current experimental and clinical findings on the usage of anti-inflammatory treatments for malignant tumors. Many studies have confirmed the cancer prevention capability of several anti-inflammatory drugs, including aspirin, celecoxib, dexamethasone, ibuprofen, piroxicam, and sulindac [245, 246]. For example, nonsteroidal anti-inflammatory drugs (NSAIDs), particularly aspirin, have prevented the development of many solid tumors by inhibiting COX2 and NF*κ*B [247–249]. Indeed, COX-2 inhibitors such as celecoxib, rofecoxib, and cisplatin have been used to prevent colorectal, lung, and breast cancers [250]. NSAID administration can reduce tumor proliferation and metastasis, as well as increase apoptosis and sensitivity to chemotherapy [251]. Additionally, perioperative NSAIDs can reduce systemic inflammation and improve the survival rate by up to 40% after the surgical removal of colorectal tumors [252].

Moreover, research has confirmed the role of dexamethasone in preventing and treating cancers. For instance, Diab et al. found that submolar concentrations of dexamethasone exert an anticancer effect in breast cancer cells [253], and Bertoli et al. showed that dexamethasone reduced the proliferation of long-term cultured leukemic cells by 38% while amplifying the cytotoxicity of doxorubicin [254]. Dexamethasone can also suppress cancer-related fatigue, nausea, and vomiting in patients undergoing chemotherapy [255]. Recently, hydrogen sulfide-releasing anti-inflammatory drugs have exhibited high efficacy and low toxicity, making them a promising option for cancer chemoprevention [256]. Thus, many anti-inflammatory drugs can not only prevent cancer occurrence but also be used as an adjunct to conventional therapy and immunotherapy. Preclinical studies have shown that anti-inflammatory agents targeting cytokines, such as TNF-*α*, IL-6, IL-8, IL-22, and IFN-*γ*, demonstrate protective effects against various types of cancer [257, 258]. Additionally, several nonsteroidal and steroidal anti-inflammatory drugs can remodel the tumor immune landscape to promote the efficacy of immune checkpoint blockade [259]. Notably, few anti-inflammatory agents have been approved by the US Food and Drug Administration for cancer treatment owing to their side effects and toxicity. Furthermore, monotherapy with anti-inflammatory drugs can lead to cell adaptability and chemotherapy resistance, fueling disease progression [256]. Therefore, substantial work is required to develop effective combination regimens in oncology.

### 5.2. Antioxidant Agents in Tumor Therapy: The Burning Question

Considering that intercellular redox imbalance is associated with tumor initiation, progression, and treatment response, the application of antioxidants in tumor therapy has gained international attention over the past 40 years. Since the 1980s, millions of people have adopted the daily consumption of vitamins E and C and selenium to prevent cancer [260, 261]. However, more recent epidemiological studies have found that the supplementation of antioxidants has a minimal preventive and therapeutic effect on cancers and may even lead to adverse effects [262–264]. In 2000, Halliwell first proposed the concept of the antioxidant paradox in *The Lancet*, which refutes the value of antioxidants in tumor treatment [265]. Currently, it remains uncertain whether antioxidant interventions should be given to oncology patients [266–268]. However, there is emerging evidence for the highly complex role of redox networks in organisms. To achieve precise and effective regulation of the intracellular redox state, antioxidant pharmacology should follow the “5R” principles, that is, “right species, right place, right time, right level, and right target” [61]. Accordingly, the antioxidant capacity of vitamins and selenium is limited as they fail to completely remove excess ROS from the human body. Interestingly, complex antioxidants and natural antioxidants exhibit superior antitumor efficacy [269–271]. Moreover, vitamin C intake below the recommended allowance leads to increased DNA oxidative damage, whereas the consumption of high-dose vitamin C can kill cancer cells [272, 273]. Several mechanisms have been proposed to illustrate the anticancer effects of high-dose vitamin C, such as induction of ROS accumulation, epigenetic reprogramming, enhanced immunotherapy efficacy, and inhibition of HIF1*α*-induced hypoxia adaptation [272, 274, 275].

According to the most recent research advances, the effect of antioxidant agents varies among different stages of cancer. First, the proper administration of antioxidants can reduce cancer incidence by scavenging the ROS that fuel cancer initiation. NAC, GSH, selenium, vitamins, polyphenolic compounds, flavonoids, and anthocyanins reportedly prevent or delay the onset of cancer by inducing the removal and detoxification of carcinogens [121, 269–271]. Dietary supplementation of fruit, vegetables, herbal medicine, and other foods rich in antioxidants (Table 4) is also recommended to prevent cancer development [276, 277]. Second, once cancerization has occurred, antioxidant supplementation often interferes with cancer treatment and patient survival by reducing ROS-dependent apoptosis [44, 268, 269]. Instead of antioxidants, prooxidants should be used to kill cancer cells in this stage. In fact, many therapeutic drugs and irradiation therapies destroy cancers by generating large-ROS doses [42, 44, 103, 217]. Moreover, engineering nanomedicines for GSH depletion can promote the efficiency of traditional therapies, which is considered a novel strategy for combating cancer [278]. Third, many studies have documented the role of antioxidant agents and Nrf2 activation in accelerating tumor metastasis; however, the related mechanisms remain unclear [119, 279, 280]. Lastly, antioxidants can also enhance therapy resistance by assisting the survival of cancer or precancer cells. For example, elevated GSH and Nrf2 levels in specific drugs may contribute to tumor progression and chemotherapy resistance [188, 267, 269, 280]. Therefore, both ROS and antioxidants have twofold effects on cancer, severely complicating the application of antioxidants in oncology therapy. Thus, precision redox-based therapy may help develop new therapeutic strategies.

## 6. Conclusions

Chronic inflammation induced by unhealthy lifestyle factors and environmental irritants can lead to many diseases, including cancer. As such, the early diagnosis and treatment of chronic inflammation will contribute to reduced cancer incidence and improve the quality of life. Oxidative stress and inflammation are closely linked to pathophysiological processes, which easily amplify each other through a feedback loop. Thus, the combined usage of antioxidant agents and anti-inflammatory drugs may be beneficial for treating chronic diseases and preventing tumorigenesis. This review highlights the crucial role of ROS in inflammation-induced tumorigenesis, whereby ROS bridge the gap between chronic inflammation and tumor development through the malignant transformation of normal cells, as well as the proliferation, survival, migration, and invasion of cancer cells (Figure 6). Notably, ROS influence tumor development in seemingly counterintuitive ways, not only fostering tumorigenesis but also killing cancer cells. Currently, the role of antioxidants in cancer treatment remains controversial; however, the consumption of dietary antioxidants is recommended to reduce the incidence of cancer.

## Figures and Tables

**Figure 1:** Intercellular ROS determines cell fate. Generally, low levels of ROS facilitate cell proliferation, high levels of ROS cause cell proliferation and malignant transformation, and toxic levels of ROS result in apoptosis and necrosis.

**Figure 2:** Cross-talk between ROS signaling and inflammatory responses. Activation of inflammatory cells results in the production of primary ROS, which contributes to the accumulation of primary cytokines by activating inflammatory transcriptional factors. In turn, primary cytokines also stimulate inflammatory cells to generate secondary ROS, leading to the further release of secondary cytokines. Once intercellular ROS reach a toxic threshold, they can induce necrotic and apoptotic cell death, ultimately causing the recruitment of more inflammatory cells.

**Figure 3:** Redox homeostasis in normal and cancer cells. The production and elimination of ROS regulate cellular redox states. Under normal conditions, cells reach redox homeostasis because their antioxidant system is sufficient to scavenge low-level ROS. Interestingly, although malignant cells generate more ROS through the activation of ETC, oncogenes, and inflammatory stimuli, an enhanced Nrf2-dependent antioxidant system contributes to cellular redox homeostasis.

**Figure 4:** ROS drives inflammation-induced genomic instability. Higher ROS cause genomic instability by inducing DNA damage and impairing DNA repair. Furthermore, cross-talk between DNA damage and inflammation leads to ROS accumulation.

**Figure 5:** ROS sources in malignant cells and their role in promoting cell proliferation. There are many sources of ROS in malignant cells, including cytokines, growth factors, NOXs, Mito-ETC, and oncogenes. Higher ROS levels facilitate the aberrant proliferation of cancer cells by regulating various signaling pathways.

**Figure 6:** ROS bridge the gap between chronic inflammation and tumor development. Chronic inflammation results in the generation of low-grade ROS in the TEM and cancer cells, contributing to tumor initiation, promotion, and progression through the regulation of various signaling pathways.

**Table 1:** Cancers, associated chronic inflammatory diseases, and their risk factors.

Cancer	Inflammatory disease	Risk factors	Reference
Lung cancer	Chronic pneumonia	Smoking, asbestos, air pollution	[17, 18]
Liver cancer	Hepatitis	Infection, alcohol, chemicals	[19–21]
Gastric cancer	Chronic gastritis	Infection, alcohol, chemicals	[22, 23]
Oral cancer	Gingivitis and periodontitis	Betel-nut, smoking, infection	[24]
Kidney cancer	Chronic nephritis	Infection, chemicals, diabetes	[25]
Skin cancer	Chronic dermatitis	Allergy, radiation, UV	[26, 27]
Pancreatic cancer	Chronic pancreatitis	Infections, alcohol, DDT, diet	[28]
Prostate cancer	Chronic prostatitis	Obesity, alcohol, infection	[29, 30]
Ovarian cancer	Ovaritis	Fertility, chemicals, obesity	[31, 32]
Bladder cancer	Chronic cystitis	Infection, chemicals, diabetes	[33, 34]
Breast cancer	Chronic mastitis	Fertility, obesity, stress	[35, 36]
Cervical cancer	Chronic cervicitis	Infection, sexuality, hygiene	[37, 38]

**Table 2:** Inflammatory factors and their classification.

Category	Proinflammatory factors	Reference
Physical factors	Radiation, UV, hyperthermia, hypothermia, trauma	[70, 71]
Chemical factors	Asbestos, heavy metals, organic toxicants, lipopolysaccharides, dust	[72–74]
Biological factors	Bacterial infection, virus infection, fungal infection	[75, 76]
Unhealthy lifestyle	Smoking, alcohol, high-calorie diet, stress, sedentary lifestyle	[77–79]
Chronic diseases	Obesity, diabetes, hyperglycemia, hyperglycemia	[80–82]
Pathologic tissues	Apoptotic cells, ischemia, hypoxia	[83, 84]
Anaphylaxis	Allergens, autoimmune diseases	[85, 86]

**Table 3:** The list of cancers linked to redox imbalance and ROS accumulation.

Cancer classification	Cancer types	Reference
Digestive cancer	Hepatocellular carcinoma, gastric cancer, bowel cancer, gallbladder cancer, pancreatic cancer	[44, 105, 117, 144]
Head and neck cancer	Oral cancer, throat cancer, thyroid cancer	[28, 145]
Urinary tract carcinoma	Ureteral cancer, bladder cancer, prostate cancer	[30, 146]
Nervous system tumor	Spinal cord tumors, astrocytomas, brain cancer	[44, 147]
Hematologic tumor	Leukemia, multiple myeloma, lymphoma	[148, 149]
Respiratory cancer	Lung cancer, bronchial carcinoid tumor	[122, 150]
Female reproductive cancer	Cervical cancer, ovarian cancer	[37, 110]
Skin cancer	Cutaneous squamous carcinoma, melanoma	[151]
Other tumors	Breast cancer, osteosarcoma	[36, 147, 152]

**Table 4:** Foods and herbal medicine rich in antioxidants.

Antioxidant agents	Foods rich in antioxidants	Reference
VA	Berries, carrot, edible plant oil, livers, nuts, eggs, fish	[281, 282]
VC	Most of the fruits and vegetables	[261, 273]
VE	Edible plant oil, dairy, meats, nuts, eggs, fish oil	[274, 283]
Flavonoids	Berries, quercetin, curcumin, soy isoflavones, baicalin, rutin	[284]
Selenium	Eggs, kidneys, oysters, konjac, alfalfa	[283, 285]
Polyphenols	Cereal brans, Resveratrol, caffeic acid, green tea, Ginkgo	[269]
Carotenoids	Carrot, broccoli, tomatoes, sweet potatoes, pumpkin	[286]
Anthocyanins	Purple cabbage, purple onion, berries, purple potato	[287]
Others	Butylated hydroxyanisole, propyl gallate	[288]

## Data Availability

No data were used to support this study.

## Abbreviations

AP-1: Activator protein-1
BER: Base excision repair
CAT: Catalase
CDKs: Cyclin-dependent kinases
CoQ: Coenzyme
COX-2: Cyclooxygenase-2
CXCL10: Chemokine ligand 10
CYP450: Cytochrome oxidase P450
DEN: Diethyl nitrosamine
EGF: Epidermal growth factor
EMT: Epithelial-mesenchymal transition
ERK: Extracellular regulated protein kinases
ETC: Electron transport chain
GPXs: Glutathione peroxidases
GSH: Glutathione
GSTs: Glutathione reductases
H_2_O_2_: Hydrogen peroxide
HIF1-*α*: Hypoxia-inducible factor-1*α*
HO-1: Hemoxygenase-1
ICAM-1: Intercellular cell adhesion molecule-1
IFN-*γ*: Interferon-*γ*
IL-6: Interleukin-6
iNOS: Inducible NO synthase
JNK: Jun N-terminal kinase
LPS: Lipopolysaccharides
MAPK: Mitogen-activated protein kinase
MCP-1: Monocyte chemotactic protein-1
MDSCs: Myeloid-derived suppressor cells
MMPs: Matrix metalloproteinases
NAC: N-acetyl-L-cysteine
NF*κ*B: Nuclear factor *κ*-B
NLRP3: NOD-like receptor protein 3
NO: Nitric oxide
NOXs: Nicotinamide adenine dinucleotide phosphate oxidases
NSAIDs: Nonsteroidal anti-inflammatory drugs
O^2-^•: Superoxide
OGG1: 8-oxoguanine glycosylase 1
ONOO-: Peroxynitrite
PGC1-*α*: Peroxisome proliferator-activated receptor coactivator 1-*α*
PKC: Protein kinase C
PMA: Phorbol 12-myristate 13-acetate
RNS: Reactive nitrogen species
ROS: Reactive oxygen species
SOD: Superoxide dismutase
STAT: Signal transducer and activator of transcription
TAMs: Tumor-associated macrophages
TGF-*β*: Transforming growth factor-*β*
TME: Tumor microenvironment
TNF-*α*: Tumor necrosis factor-*α*
VEGF: Vascular endothelial growth factor
4-HNE: 4-Hydroxynonenal
8-OHdG: 8-Hydroxydeoxyguanosine.
